# Evaluation of the Antibacterial Effect of Xylene, Chloroform, Eucalyptol, and Orange Oil on *Enterococcus faecalis* in Nonsurgical Root Canal Retreatment: An Ex Vivo Study

**DOI:** 10.1155/2022/8176172

**Published:** 2022-09-23

**Authors:** Mohsen Aminsobhani, Hassan Razmi, Fatemeh Hamidzadeh, Arvin Rezaei Avval

**Affiliations:** ^1^Department of Endodontics, Faculty of Dentistry/Dental Research Center, AJA and Tehran University of Medical Sciences, Tehran, Iran; ^2^Department of Endodontics, Faculty of Dentistry, Tehran University of Medical Sciences, Tehran, Iran

## Abstract

**Objectives:**

The present ex vivo study is aimed at evaluating the antibacterial efficacy of chloroform, eucalyptol, orange oil, and xylene against *E. faecalis* biofilm during nonsurgical root canal retreatment.

**Materials and Methods:**

Eighty single-rooted teeth were instrumented. The samples were autoclaved, infected with *E. faecalis* for 4 weeks, and obturated with gutta-percha. Then the teeth were randomly assigned to 4 groups (*n* = 20): (1) chloroform, (2) eucalyptol, (3) orange oil, and (4) xylene. In all of the groups, gutta-percha removal was conducted according to the same protocol although the solvent used in each group was different. Bacterial samples were collected after gutta-percha removal and following additional apical enlargement. Intergroup and intragroup analyses were conducted using one-way ANOVA combined with the post hoc Tukey test and the paired-sample *t*-test, respectively. Statistical significance was set to 0.05.

**Results:**

All of the groups showed more than 99% bacterial load reduction. The least bacterial load after gutta-percha removal was observed in the chloroform group (*p* < 0.001). The orange oil group showed a significantly lower bacterial load compared to the eucalyptol group (*p* = 0.001), while it was not different from the xylene group (*p* = 0.953). The xylene group also had a significantly lower bacterial load compared with the eucalyptol group (*p* = 0.017). After apical enlargement, the chloroform group had a significantly lower bacterial load compared to the other groups. The comparison of bacterial load values before and after apical enlargement in the chloroform and eucalyptol groups showed a statistically significant difference (*p*_choloroform_ = 0.011, *p*_eucalyptol_ = 0.001).

**Conclusion:**

Chloroform was the most effective solvent in terms of antimicrobial activity against *E. faecalis* followed by orange oil and xylene, which were not significantly different though, and eucalyptol. All of the solvents showed more than 99% bacterial load reduction. Chloroform and xylene revealed to be associated with favorable antibiofilm activity among the examined solvents.

## 1. Introduction

Posttreatment persistent periapical infections occur mainly due to intraradicular infection, extraradicular infection, foreign body reaction, cysts (especially those containing cholesterol crystals), and fibrous scar tissue healing [1]. Despite several possible nonmicrobial etiologies, root canal treatment failure is mainly attributed to the persistence of microorganisms in the apical part of previously-treated teeth [1, 2].

Although primary endodontic infections are polymicrobial with Gram-negative anaerobic rods reported as the dominant species, secondary infections are associated with one or more bacterial species, i.e., secondary infections are limited to a narrower spectrum of bacteria [2–5]. *Enterococcus faecalis* has been isolated from not only necrotic cases but also previously-treated ones. Previous observations had shown that it constitutes a small part of the untreated cases' microbial profile. However, evidence suggests that *E. faecalis* plays a key role in forming persistent lesions after root canal treatment [1, 6]. Along with the association of root canal treatment failures with the presence of this species, the high potential to tolerate the starvation phases and its capability to survive in the root canal as a single organism or as a major component of the microbial flora may testify its major contribution to secondary root canal infections. Besides, biofilm formation has been proved to play an important role in enterococcal infection of root canal [7, 8].

*E. faecalis* is a Gram-positive cocci that can be in a single form, in pairs, or short chains. It is a facultative anaerobe that is able to withstand harsh conditions such as high alkalinity and high salt concentrations. Enterococcus species are capable to live in large numbers in the intestinal tract and in most cases, do not harm their host. These bacteria are also present in smaller numbers in the female genital tract and oral cavity. They use carbohydrates, glycerol, lactate, malate, citrate, arginine, and keto-acids as sources of metabolic fuel [9].

Treatment of *E. faecalis* infections is challenging due to the high microbial resistance observed in some cases [10]. The prevalence of *E. faecalis* in the obturated root canals has been reported from 24% to 77%. The wide range of reported findings might be due to different identification techniques, geographical differences, or sample sizes [3–5, 11–19]. While the polymerase chain reaction (PCR) test is suggested as a more predictable identification technique, most of the studies have used microbial culture techniques [20, 21]. PCR-based studies have reported its prevalence from 67% to 77%, which was higher than the prevalence of 24% to 70% reported by culture-based studies [18]. *E. faecalis*, besides several aforementioned virulence factors, can attach to host cells, change host responses, and suppress the lymphocytes' activity [18, 22, 23]. Considering the substantial contribution of this microorganism to the root canal treatment failure and the high treatment resistance reported by several studies, a combination of disinfecting procedures might result in more satisfying outcomes. Increasing the size of the apical portion of the canal, removing the smear layer, and using disinfection protocols to penetrate the dentinal tubules were the most highlighted strategies taken to overcome such a microbial challenge [24, 25]. While some studies have mentioned that 3-6% sodium hypochlorite, when used in high volume and sufficient contact time, can remove *E. faecalis* from the canal, others still do not agree with the idea that sodium hypochlorite can eradicate this species [25]. Smear layer removal protocols [26], several irrigant activation techniques [27], and several intracanal medicaments [28] have been suggested to overcome *E. faecalis*; however, it remains a challenge, particularly in nonsurgical root canal retreatments.

Nonsurgical root canal retreatment includes removal of root canal filling materials, which is nowadays mostly gutta-percha. Complete removal of the filling material is usually a time-consuming and challenging process, but an essential for proper access to the root canal system and ideal disinfection [29]. There are different ways to remove gutta-percha and sealer from the root canal system, including the application of heat or different solvents to soften the material followed by using hand files, burs, and automatic engine-driven instruments [30].

Chloroform, orange oil, xylene, halothane, and eucalyptol have all been introduced as gutta-percha solvents [31]. Chloroform is the most common gutta-percha solvent because it dissolves gutta-percha efficiently and has been associated with high treatment success rates [32]. Chloroform and eucalyptol have been used as gutta-percha solvents since 1850 [33]. The efficacy and advantages of chloroform as a gutta-percha solvent during retreatment have been well established. However, it is toxic and has been shown to have carcinogenic effects [32]. Considering the high probability for a gutta-percha solvent to come into contact with periodontal and periapical tissues during the treatment procedure [34], the use of chloroform has been forbidden in some countries [32]. Xylene and eucalyptol are currently the most common solvents used by dentists [31]. Xylene is known to be the most effective gutta-percha solvent [35], while its toxicity as well as negative effects on the central nervous system have been proven [36]. Eucalyptol can be used as an alternative substance that does not have the aforementioned side effects [36], although studies have shown that it dissolves gutta-percha with lower efficacy compared to chloroform and xylene at room temperature, but its efficacy increases in higher temperatures [31]. Orange oil, as another gutta-percha solvent, has been suggested to be equal to xylene in terms of dissolving efficacy [36].

Few studies have been performed on the possible antibacterial effects of gutta-percha solvents. A previous ex vivo study that investigated the antimicrobial efficacy of chloroform suggested that microbial load would decrease significantly when chloroform is applied as gutta-percha solvent [37]. Another study compared the antimicrobial efficacy of chloroform with orange oil and eucalyptol when applied on infected bovine dentin blocks and concluded that all of these solvents have favorable antimicrobial characteristics against *E. faecalis.* While chloroform was the most effective solvent, orange oil showed higher antimicrobial potential compared to eucalyptol [38]. However, a recent in vitro study comparing turpentine oil, eucalyptus oil, orange oil, chloroform, and xylene with regard to their antibacterial potential suggested that after turpentine oil, eucalyptus oil was the most effective solvent followed by orange oil, chloroform, and xylene, respectively [39]. However, it is important to consider that when it comes to the real clinical context, a combination of factors contributes to the complexity of the treatment of such cases, e.g., efficacy of the solvent in gutta-percha removal combined with its antimicrobial potential and presence of biofilm-form of the microorganism. To the best of our knowledge, the antimicrobial potential of the aforementioned solvents has not been examined on the *E. faecalis* biofilm when recruited in a routine nonsurgical root canal retreatment procedure. Thus, the present study is aimed at investigating the antimicrobial potential of chloroform, orange oil, eucalyptol, and xylene against *E. faecalis* in nonsurgical root canal retreatments.

## 2. Materials and Method

A total of 80 single-rooted human teeth with mature apex, extracted due to periodontal problems or orthodontic treatment plans, were collected. The study protocol was approved by the Tehran University of Medical Sciences Ethical Committee (IR.TUMS.DENTISTRY.REC.1400.133). The presence of only one canal was confirmed by radiography from two aspects. The teeth were immersed in 5.25% sodium hypochlorite for 30 minutes to remove residual tissue and debris on the root surface. After access cavity preparation, a #10 K file was inserted into the canal till it was seen from the apical foramen. The working length was determined by subtracting one millimeter from this length. Mechanical canal preparation was performed using SP1 Gold rotary system (SP1, Fanta-dental, China) S1, S2, F1, F2, and F3 rotary files. In all cases, after using each file, the canal was irrigated with 1 ml of 5.25% sodium hypochlorite solution using 30-gauge side-vented needles (Tribest, China). Apical patency was established with a #10 K file. Teeth were autoclaved at 121°C for 30 minutes (15 psi). Each tooth was placed into a 1.5 ml micro tube (Eppendorf Safe-Lock Tubes, Eppendorf, Dubai, UAE) containing 1 ml of sterile water. The vials were sealed and incubated at 37°C for 2 days to rehydrate the teeth. The canal and pulp chamber of all teeth were filled with the pure *E. faecalis* suspension (ATCC 29212) cultured in Brain Heart Infusion (BHI) medium. All teeth were incubated at 37°C for 4 weeks. At 72-hour intervals, micro tubes were refilled with fresh BHI medium. During fluid replacement, random sampling of the canal fluid was taken to confirm the positive culture of *E. faecalis.* After the incubation period, a random sample was selected and processed to confirm the presence of *E. faecalis* biofilm on the root canal walls by the Scanning Electron Microscopy. Then the teeth canals were dried with sterile paper cones and obturated using lateral compaction technique. Master gutta-percha cones were selected based on the Master Apical File (MAF) size which was either #40 or #45. The sealer used for root canal obturation was GuttaFlow 2 (Roeko, Coltene, Switzerland). Finally, the excessive gutta-percha was cut at the CEJ level and packed into the canal. Then, the teeth were kept for another 6 weeks in micro tubes filled with BHI.

### 2.1. Gutta-Percha Removal

After 6 weeks, samples were assigned to 4 groups (*n* = 20), and in each group, one of the solvents, including chloroform (Golchadent, Iran), eucalyptol (Cerkamed, Poland), orange oil (Moksha Life Style Products, India), and xylene (Merck, Germany), were used during the gutta-percha removal procedure. In order to remove gutta-percha, these steps were followed: (1) the pulp chamber was filled with 2 or 3 drops of a solvent, (2) a #2 gates-glidden drill (MANI, Japan) was used for 2 to 3 mm penetration into the softened gutta-percha with least pressure, (3) the unfilled part of the canal was filled with 2 or 3 drops of the solvent, (4) #35 and #40 H files were used to penetrate the gutta-percha till the H file reached the WL, (5) excessive gutta-percha masses on the canal walls were tried to be pulled out by H files, (6) the remaining gutta-percha was removed from the canal walls by wicking technique, i.e., the canal was filled with solvent and after 30 seconds the canal was dried using paper points (Meta, Seoul, Korea). This step was repeated until paper points were free of gutta-percha residues. First bacterial sampling was conducted at this time point, and (7) the canal was instrumented with an F4 rotary file to the WL, and the second bacterial sampling was conducted.

### 2.2. Sample Collection and Bacterial Load Assessment

To collect bacterial samples, a standard method was recruited: the empty dry canal of the tooth was filled with saline as a transport medium. A #15K file was introduced into the canal within 1 mm of working length and circumferentially pulled along the canal walls for 10 seconds. Three consecutive paper points were used to collect the sample. The paper points were placed separately in the Eppendorf tubes containing 1 ml BHI. This procedure was conducted once after gutta-percha removal (step 6) and once after apical enlargement (step 7).

All samples were vortexed for ten seconds and tenfold dilutions (10^−1^ to 10^−10^) were prepared in saline. 100 *μ*l of each sample dilution was spread plated onto BHI agar plates, incubated at 37°C for 48 hours, and colony-forming units (CFUs) per 1 ml were counted (Figure 1).

### 2.3. Statistical Analysis

95% confidence intervals for each group's bacterial load at each study phase were calculated. Data were analyzed in SPSS 26.0 (IBM Corporation, NY, USA). After confirming the normality of the distribution of the data, one-way ANOVA combined with post-hoc Tukey's tests were used to compare different solvents, and the results were reported as intergroup analysis. Intragroup analysis was conducted using the paired-sample *t*-test to compare the bacterial load at each phase of the study in each experimental group. The significance level was set to 0.05.

## 3. Results

The biofilm formation was confirmed using the Field Emission Scanning Electron Microscopy of the intracanal surface of a random sample 4 weeks after bacterial culture (Figure 2).

The results of the antimicrobial efficacy of each solvent are presented in Table 1. All of the groups showed more than 99% bacterial load reduction not only after gutta-percha removal but also after apical enlargement. Bacterial survival rates in each group at each phase of the study are reported in Table 2.

### 3.1. Intergroup Analysis

Intergroup statistical analysis of the after-gutta-percha-removal data showed that bacterial load was significantly lower in the chloroform group (*p* < 0.001). The orange oil group showed a significantly lower bacterial load compared to the eucalyptol group (*p* = 0.001), while it was not different from the xylene group (*p* = 0.953). The xylene group also had a significantly lower bacterial load compared with the eucalyptol group (*p* = 0.017). All of the groups showed significantly lower bacterial load compared to the control group at this phase (*p* < 0.001). Percentage of bacterial load reduction after gutta-percha removal revealed that chloroform was significantly more effective than eucalyptol and orange oil (*p* < 0.001). Orange oil was significantly more effective than eucalyptol (*p* = 0.002).

Intergroup statistical analysis of the after-apical-enlargement data suggested that only the chloroform group had significantly lower bacterial load compared to the other groups, while there was no difference between other groups at this phase. The percentage of bacterial load reduction after apical enlargement again suggested chloroform as the most effective solvent (*p* < 0.001), while the others were statistically the same in terms of antimicrobial efficacy (*p* > 0.05).

### 3.2. Intragroup Analysis

Before and after apical enlargement bacterial load logarithmic values are illustrated in Figure 3. Comparing the before and after apical enlargement microbial load in the chloroform and eucalyptol groups showed statistically significant differences (*p*_choloroform_ = 0.011, *p*_eucalyptol_ = 0.001), while the same comparison did not reveal a significant difference in the other groups. The same comparison did not show a statistically significant difference in the control group.

In Figure 4 representative FE-SEM images of each group of the study after the retreatment procedure are presented. SEM images suggested that chloroform and xylene had higher antibiofilm activity potential than other studied solvents.

## 4. Discussion

The present study focused on the antibacterial potential of two synthetic gutta-percha solvents, chloroform and xylene, and two organic gutta-percha solvents, orange oil and eucalyptol, on *E. faecalis* biofilm during nonsurgical root canal retreatment procedure in ex vivo models. The results suggested that all of the solvents could reduce the microbial load by more than 99% not only after gutta-percha removal but also after further apical enlargement. Although chloroform as a synthetic solvent was superior to the other solvents in terms of antimicrobial efficacy, orange oil showed favorable results, which were comparable with xylene. Eucalyptol ranked as the least efficient solvent with regard to antimicrobial effects.

The results of the present study suggested that chloroform was significantly superior to the other solvents, either organic or synthetic ones. In this group, even negative cultures were observed. This finding was in agreement with Edgar et al. [37] and Martos et al. [38] findings, which reported that chloroform had high antimicrobial potential against *E. faecalis* and it was reported to be able to eradicate *E. faecalis*. Xylene was similar to orange oil, while they were both superior to eucalyptol. However, Hunter et al. in a previous study have suggested that chloroform was similar to eucalyptol and orange oil [34]. Martos et al. have reported that orange oil was more effective than eucalyptol when the contact time of the solvent with bacterial biofilm increased [38], which was in agreement with the present study's findings. However, another study suggested that orange oil was not effective against *E. faecalis* while eucalyptol had antimicrobial potential against this microorganism [40]. Subbiya et al. have reported that xylene does not have any antimicrobial effects against *E. faecalis* [41], while the present study and another recent one [39] observed antimicrobial properties for this solvent. The variable findings across studies might be attributed to the methodological diversity among them.

Some strains of a cultivable species can be uncultivable. It has been mentioned as a survival strategy for some bacteria, i.e., they have a state called “Viable But Not Cultivable” (VBNC) in which they cannot be detected by conventional culturing methods. Such a strategy has been described in some Gram-negative species but recently also for *E. faecalis*. These strains must be detected using Polymerase Chain Reaction (PCR) [42]. In the present study, the antibacterial effect of solvents only on cultivable strains was evaluated; thus, the results should be interpreted with caution, i.e., the 99% bacterial load reduction refers to the reduction of the load of cultivable strains in particular.

Eucalyptol, extracted from the leaves of *Eucalyptus globulus*, has been associated with antimicrobial and anti-inflammatory properties. Such findings about this solvent have been mainly attributed to 1,8-cineole, which is known as the main constituent of eucalyptol [43, 44]. The low dissolution ability of this solvent, the main disadvantage of it, which was reported in the previous studies could be overcome by increasing the temperature [31]. However, in the present study, it was recruited at room temperature and was associated with satisfying results although not comparable to the synthetic solvents.

Orange oil, extracted from the peel of *Citrus sinensis*, is mainly composed of D-limonene. The better dissolution ability of this solvent has made it a valuable alternative to synthetic solvents. This compound exerts its antimicrobial effects by interfering with ATP synthesis, bacterial cell homeostasis, and bacterial membrane permeability [45–47]. This solvent is biocompatible and clinically safe [39]. In the present study, orange oil was comparable to xylene in terms of antimicrobial activity.

Important characteristics other than favorable antimicrobial activity, a clinician may consider when choosing one solvent among the alternatives are dissolution ability, biocompatibility, cytotoxicity, carcinogenicity, better odor, and availability. Although synthetic solvents are reported to be more effective in terms of dissolution ability and antimicrobial effects, they are associated with less biocompatibility and might have hazardous effects on host tissues [39]. Chloroform was banned by the U.S. Food and Drug Administration in 1976 due to the potential adverse effects on the host tissues [37, 48]. Although several studies have reported xylene as the most efficient solvent, unsafety and unfavorable odor are the main challenges with this solvent [39]. Although essential oils, e.g., eucalyptol and orange oil, have been reported to be less effective in gutta-percha dissolution, they have been associated with favorable antimicrobial effects even comparable to the synthetic solvents'. Considering the biocompatibility, favorable odor, high antimicrobial activity, less cytotoxicity, and nonmutagenicity of organic solvents, they seem to be applicable alternatives to the synthetic ones.

The second sample, which was taken after further instrumentation of the apical third of the canal, revealed that the chloroform group had the least bacterial load and the others were not significantly different. The fact that all of the groups had more than 99% load reduction after further instrumentation suggests that all of the solvents were able to penetrate the infected dentine and affect bacterial biofilm in the deeper areas; however, chloroform proved to be associated with more satisfying results.

Antibiofilm activity of solvents was evaluated using FE-SEM images. The present study's results suggested that chloroform had the highest antibiofilm activity among the solvents, this finding corroborated a previous study's [38] findings which suggested that chloroform had the highest antibiofilm activity potential against *E. faecalis* in comparison with orange oil and eucalyptol. Xylene was also associated with favorable antibiofilm activity. Organic solvents examined in the present study failed to affect *E. faecalis* biofilm.

The present study tried to examine gutta-percha solvents' antimicrobial activity potential against *E. faecalis*, one of the most important challenges of nonsurgical root canal retreatments, in an ex vivo model. Recruiting ex vivo models, unlike previous studies that examined the antimicrobial activity of these solvents in the absence of other contributing factors, might provide the clinicians with more realistic findings. In a clinical setting, a combination of contributing factors may compromise the antimicrobial potential of a specific solvent, as the low dissolution ability of a solvent might compromise infected gutta-percha removal which leads to higher observed microbial load after the treatment or the biofilm form of the microorganism, which is known for its treatment-resistance, might be less susceptible than the planktonic form and have been mainly associated with treatment failures. All of these contributing factors were considered in the present study, while they were not simulated in the previous ones. While the study results indicated that solvents had favorable antimicrobial potential against the planktonic form of *E. faecalis*, only the chloroform and xylene groups were associated with favorable antibiofilm activity. On the other hand, the detection technique used in the present study was culturing which is unable to detect all forms of *E. faecalis*, i.e*.,* the reported bacterial load reduction is limited specifically to the culturable species. In the present study, in order to standardize the methodology, single-rooted teeth were recruited as the study samples, while multirooted teeth are associated with more challenges in gutta-percha removal and root canal disinfection. As an ex vivo study in which the tooth was evaluated separately not in relation to its supporting structures and the whole body, results should be interpreted with caution. Future studies may focus on the other organic solvents with higher dissolution ability and favorable antimicrobial activity or making some modifications to the examined ones to make them more satisfying in a clinical setting. In vivo studies are necessary to evaluate short-term and long-term outcomes associated with the use of different gutta-percha solvents during nonsurgical root canal retreatment.

## 5. Conclusion

Within the limitations of this study, chloroform proved to be the most effective solvent in terms of antimicrobial activity against *E.faecalis* followed by orange oil and xylene, which were not significantly different though, and eucalyptol. Chloroform and xylene revealed to be associated with favorable antibiofilm activity among the examined solvents. All of the solvents showed more than 99% bacterial load reduction which sounds like good news. In other words, the examined solvents contribute to the root canal disinfection procedure, which is a challenge in nonsurgical root canal retreatments, besides their own responsibility in root canal filling materials removal.

## Figures and Tables

**Figure 1:** A flow chart of the experimental process.

**Figure 2:** *E. faecalis* biofilm formation confirmed by the Scanning Electron Microscopy with 3Kx (a) and 20Kx (b) magnification.

**Figure 3:** Mean log CFU of each experimental group at each study phase.

**Figure 4:** Representative FE-SEM images of each group of the study after treatment with gutta-percha solvents.

**Table 1:** Load of *E. faecalis* after gutta-percha removal and after apical enlargement for each experimental group (95% CIs are reported).

Solvent	After gutta-percha removal (CFUs/ml)	After apical enlargement (CFUs/ml)
Chloroform	4.24-19.89^Aa^	1.14-4.25^Ba^
Eucalyptol	2345.85-4301.30^Ab^	197.79-1145.51^Bb^
Orange oil	471.09-1480.47^Ac^	396.28-2619.99^Ab^
Xylene	207.21-1540.64^Ac^	95.72-741.14^Ab^

∗Different capital letters (A and B) in the same line indicate statistical significance (*p* < 0.05). ∗∗ Different small letters (a, b, and c) in the same column indicate statistical significance (*p* < 0.05).

**Table 2:** Mean of the bacterial survival rates in different experimental groups at each phase of the study.

Solvents	After gutta-percha removal survival rate	After apical enlargement survival rate
Chloroform (*n* = 20)	1.6∗10^−6^	1.41∗10^−6^
Eucalyptol (*n* = 20)	2.24∗10^−4^	2.88∗10^−5^
Orange oil (*n* = 20)	5.89∗10^−5^	6.17∗10^−5^
Xylene (*n* = 20)	3.98∗10^−5^	1.62∗10^−5^

## Data Availability

The data supporting the findings of the present study are available from the corresponding author upon request.
